# Inhibition of *α*-Amylase, *α*-Glucosidase, and Lipase, Intestinal Glucose Absorption, and Antidiabetic Properties by Extracts of *Erodium guttatum*

**DOI:** 10.1155/2022/5868682

**Published:** 2022-08-17

**Authors:** Kaoutar Benrahou, Hanae Naceiri Mrabti, Abdelhakim Bouyahya, Nour Elhouda Daoudi, Mohamed Bnouham, Hicham Mezzour, Shafi Mahmud, Mohammed Merae Alshahrani, Ahmad J. Obaidullah, Yahia Cherrah, My El Abbes Faouzi

**Affiliations:** ^1^Laboratory of Pharmacology and Toxicology, Bio Pharmaceutical and Toxicological Analysis Research Team, Faculty of Medicine and Pharmacy, Mohammed V University in Rabat, BP 6203, Rabat, Morocco; ^2^Laboratory of Human Pathologies Biology, Faculty of Sciences, Mohammed V University in Rabat, Rabat, Morocco; ^3^Laboratory of Bioresources, Biotechnology, Ethnopharmacology, and Health, Faculty of Sciences Mohammed First University, Oujda, Morocco; ^4^Laboratoire d'analyses Biologiques, Angle 498, Avenue des FAR Larache, CP 92000, Larache, Morocco; ^5^Division of Genome Sciences and Cancer, The John Curtin School of Medical Research, and The Shine-Dalgarno Centre for RNA Innovation, The Australian National University, Canberra, Australia; ^6^Department of Clinical Laboratory Sciences, Faculty of Applied Medical Sciences, Najran University, Najran 61441, Saudi Arabia; ^7^Drug Exploration and Development Chair (DEDC), Department of Pharmaceutical Chemistry, College of Pharmacy, King Saud University, Riyadh 11451, Saudi Arabia; ^8^Department of Pharmaceutical Chemistry, College of Pharmacy, King Saud University, Riyadh 11451, Saudi Arabia

## Abstract

*Erodium guttatum* is widely used in traditional medicine to treat various diseases, including diabetes. In this study, we evaluated *in vitro* inhibitory activity of extracts of *E. guttatum* on *α*-amylase, *α*-glucosidase, and lipase and then studied *in vivo* using different animal models. The results showed that the aqueous and alcoholic extracts of *E. guttatum* significantly inhibited digestive enzymes. The extracts of *E. guttatum* significantly reduced postprandial hyperglycemia after starch loading in normal rats. Additionally, extracts of *E. guttatum* significantly decrease the intestinal absorption of D-glucose. However, the methanolic extract of *E. guttatum* showed remarkable antidiabetic activity compared to the aqueous and ethanolic extracts of *E. guttatum*. In addition, the extracts significantly reduced blood sugar levels in albino mice and hematological and biochemical profiles. Therefore, the results of this study show that the extracts of *E. guttatum* have antidiabetic effects and could therefore be suggested in the management of type 2 diabetes.

## 1. Introduction

Type 2 diabetes, in other words, noninsulin-dependent diabetes mellitus, is a major health problem. The etiology of type 2 diabetes is multiple, including genetic, epigenetic, environmental, and unhealthy lifestyle factors [1]. It is linked to metabolic disorders or damage to peripheral tissues. The main pathogenic features of T2DM include damage to pancreatic cells and insulin sensitivity of organs, which lead to defective insulin secretion and resistance to blood sugar [2]. In contrast, the management of postprandial blood sugar is necessary for the early treatment of diabetes and the reduction of chronic complications [3]. Among the therapeutic strategies currently discussed to manage hyperglycemia and hyperlipidemia, this will depend on the inhibition of digestive enzymes to delay the absorption of carbohydrates and lipids and consequently the decrease in plasma levels of carbohydrates and lipids in the blood [4]. However, complex polysaccharides are hydrolyzed into oligosaccharides by the *α*-amylase enzyme, and then they are cleaved by the digestive enzymes, in particular *α*-glucosidase, into simple monosaccharides easily absorbed at the level of the intestinal border [5]. In addition, the main function of pancreatic lipase is the degradation of triacylglycerides into glycerol and free fatty acid [6]. However, blocking these enzymes will help prolong digestion time by slowing breakdown, causing reduced absorption and elevated postprandial blood sugar [7]. The antidiabetic drugs used have harmful effects or unwanted contraindications and cannot restore normal blood sugar homeostasis. This is why various enzyme inhibitors have been developed and drawn from plant resources [8]. Also, numerous ethnobotanical studies carried out in Morocco showed that medicinal plants are frequently used with a percentage of 55 to 90% depending on the region [9].

The genus *Erodium* is made up of around 74 species, distributed all over the continents with the exception of the Antarctic [10], very widespread in the Mediterranean region, with around 63 species, while other regions contain only a few native species, such as North America, South America, Australia, and Asia [11].

It has been reported that *Erodium* species are used in folk medicine to treat various diseases such as hemorrhage, dermatological, gastrointestinal disorders, indigestion, inflammatory diseases, diabetes, constipation, eczema, and as a carminative agent. Also, *Erodium* leaves have been used for the preparation of salads, omelets, sandwiches, sauces, soups, and certain food products [12].

For this, our study was carried out to the evaluation of root extracts of *E. guttatum* on the antidiabetic activity *in vitro* on the digestive enzymes *α*-amylase, *β*-glucosidase, and pancreatic lipase, to the study of tolerance to starch (OSTT), and the mode of action of the extracts on the intestinal absorption of D-glucose by the intestinal infusion method in normal rats. For the *in vivo* study in mice made diabetic by a high-fat diet and streptozotocin (HFD-STZ), by monitoring body weight and blood sugar levels as well as by analyzing certain hematological and biochemical parameters.

## 2. Materials and Methods

### 2.1. Standards and Reagents

*α*-Glucosidase from *Saccharomyces cerevisiae*, *α*-amylase from *Bacillus licheniformis,* porcine pancreatic lipase, p-nitrophenyl-*α*-D-glucopyranoside, 4-nitrophenyl butyrate, phlorizin hydrate, acarbose, orlistat, and streptozotocin were purchased from Sigma-Aldrich, USA.

### 2.2. Plant Material

The roots of *E. guttatum* were collected in February 2018 from the province of Oujda, Northern Morocco, from the latitude of 34°40′55.06″ N and a longitude of 1°54′0.56″ W, at 549 m of 250 mm of average annual rainfall. The specimen was identified by the botanist Mohammed Fennane and was deposited at the Botanical Herbarium of the Scientific Institute of Rabat under the reference number RAB 110970. The roots of *E. guttatum* were dried in the shade and then ground, and the ground material obtained was stored in a dry place and protected from humidity and light.

### 2.3. Preparation of the Plant Extracts

#### 2.3.1. Preparation of Aqueous Extract

For the preparation of the aqueous extract, 30 g of the plant material was extracted by the infusion method for 1 hour and left to cool. Subsequently, the mixture was filtered and the resulting filtrate was evaporated under vacuum at 50°C using a rotary evaporator. The extract obtained was frozen and then lyophilized to remove traces of water [13].

#### 2.3.2. Preparation of Alcoholic Extracts

For the preparation of the ethanolic and methanolic extracts, a quantity of 30 g of plant material was macerated, respectively, with 300 mL of ethanol and of methanol for 48 hours with mechanical stirring. The extracts were then filtered and evaporated using a rotary evaporator at 40°C [13].

### 2.4. Antihyperglycemic Activity

#### 2.4.1. *In Vitro* Test on the Activity of *α*-Amylase

The inhibition of *α*-amylase was tested by the starch-iodine method described by Chakrabarti et al. [14] with a few modifications. Indeed, 250 *μ*L of each sample was mixed with 100 *μ*L of the phosphate buffer solution (20 mM, PH 6.9) containing the enzyme (*α*-amylase). Then the reaction mixture was incubated at 37°C for 10 min, after which 600 *μ*L of starch (1%) was added and the mixture was reincubated at 37°C for 10 min. At the end, 25 *μ*L of the HCl solution and 100 *μ*L of the iodine solution were added. The reading was carried out by a spectrophotometer at 630 nm.

The results were expressed as percentage inhibition and calculated using the following formula:

(1) $$\begin{array}{c} \text{inhibition}\left(\%\right):\left(1-\left(\frac{{\text{OD}}_{\text{Testsample}}}{{\text{OD}}_{\text{Control}}}\right)\right)\times 100. \end{array}$$

#### 2.4.2. *In Vitro* Test on the Activity of *α*-Glucosidase

The *α*-glucosidase inhibition test was determined by the method described by Kee et al. [15]. P-nitrophenyl-*α*-D-glucopyranoside (*ρ*NPG) was used as the substrate. The *ρ*NPG was hydrolyzed by *α*-glucosidase to release the *ρ*-nitrophenyl. Acarbose was used as a positive control. In brief, 150 *μ*L of extract solution was mixed with 100 *μ*L of enzymatic solution (*α*-glucosidase). The reaction mixture was incubated for 10 minutes, then 200 *μ*L of substrate *ρ*-nitrophenyl-*α*-D-glucopyranoside (pNPG) was added, thereafter a further incubation was carried out for 30 minutes, and at the end, 1 ml of 0.1 M Na_2_CO_3_ was added to stop the reaction. The reading was carried out by a spectrophotometer at 405 nm.

The percentage of inhibition was calculated according to the following formula:

(2) $$\begin{array}{c} \text{inhibitory activity}\left(\%\right):\left[\frac{\left.{\text{OD}}_{\text{Control}}-{\text{OD}}_{\text{Test sample}}\right.}{{\text{OD}}_{\text{Controle}}}\right]\times 100. \end{array}$$

#### 2.4.3. *In Vitro* Test on the Activity of Lipase

The lipase inhibition test was evaluated by the method of Hu et al. [16] with some modifications. Orlistat was used as a reference compound. In brief, 150 *μ*L of the sample or orlistat was mixed with 500 *μ*L of the lipase enzyme (2 U) dissolved in Tris-HCl buffer (1 mM, pH8). The reaction mixture was incubated for 30 minutes at 37°C, then 450 *μ*L of 1 mM 4-nitrophenyl butyrate substrate was added and then reincubated for 30 minutes at 37°C.

The absorbance was measured at 405 nm. The percent lipase inhibition was calculated by the following formula:

(3) $$\begin{array}{c} \text{inhibition}\left(\%\right)=\left[\frac{\left(Ac-Acb\right)-\left(As-Asb\right)}{Ac-Acb}\right]\times 100, \end{array}$$

where Ac refers to the absorbance of the control, Acb refers to the absorbance of the control blank, As is the absorbance of the sample, and Asb is the absorbance of the blank sample.

#### 2.4.4. Experimental Animals

Male and female Wistar rats weighing 150–250 g were used in the experiments. The animals were kept in cages at the Rabat Faculty of Medicine and Pharmacy. They were kept under standard conditions and fed a standard diet and water. The research was carried out according to the principles described in the 8th edition of the “Guidelines for the Care and Use of Laboratory Animals” of the National Academy of Sciences (National Research Council of the National Academy of Sciences, 2011). Every effort has been made to reduce the suffering and the number of animals. Ethics approval was obtained from Mohammed V Rabat University in Rabat.

#### 2.4.5. Oral Starch Tolerance in Normal Rats

In this experimental study, the antidiabetic effect of *E. guttatum* extracts was evaluated according to the protocol described by Beejmohun et al. [17]. Rats were divided into six groups consisting of five rats each (*n* = 6). The animals were fasted overnight for 18 h but had free access to water. The control group received the vehicle (distilled water); the negative control group received vehicle (starch); the control positive group received acarbose at 50 mg/kg; and three other groups were treated with the aqueous, ethanolic, and methanolic extracts of *E. guttatum* at 150 mg/kg by gavage (*p.o*). Thirty minutes later, all the animals were loaded with starch orally at a dose of 2.5 mg/kg. Blood was collected from the tail vein before (*t* = 0), and at 30, 60, 90, and 120 min after starch administration.

#### 2.4.6. Intestinal Perfusion *In Situ*

The study of intestinal absorption in situ is carried out according to the protocol described by Ouassou et al. [18]. In order to assess the effect of aqueous, ethanolic, and methanolic extracts obtained from *E. guttatum* on glucose uptake at the jejunal segment in normal fasting rats for 36 h and anesthetized by intramuscular injection with sodium pentobarbital (50 mg/kg). The three extracts at a dose of 200 mg/kg were added to the physiological solution of (g/L) 7.37 NaCl, 0.2 KCl, 0.065 NaOH_2_ PO_4_, 2H_2_O, 0.213 MgCl_2_, 6H_2_O, 0.6 NaHCO_3_, and 1.02 CaCl_2_ and 1 g of added glucose, at pH 7, 5. The jejunal segment (10 cm) was perfused with a peristaltic pump at 0.53 mL/min for 1 hour.

Five groups of Wistar rats weighing 150–250 g were used: one group as a positive control perfused with the perfusion solution; one group as a negative control received the solution containing the standard inhibitor of D-glucose (Phlorozin 0.1 mM); and the other three groups received the solution of the three extracts. The perfusate was collected and the glucose concentration was measured using a commercial kit (glucose oxidase peroxidase, SGM Italia) and the length of the perfused segment was measured and the amount of glucose absorbed was expressed in mg/10 cm/h.

### 2.5. *In Vivo* Antidiabetic Activity

#### 2.5.1. Experimental Protocol

Swiss male and female mice weighing 20–30 g were subjected for 1 month to a diet high in fat containing standard dietary carbohydrates 50%, protein 18%, fat 30%, and salt and vitamin 2% [19]. After 4 weeks, diabetes was induced by intraperitoneal injection of streptozotocin (100 mg/kg) dissolved in a citrate buffer solution (0.1 M, pH 4.5). After five days, blood sugar was measured at the level of the tail vein. Mice with blood sugar levels above 1.26 g/L were considered type 2 diabetic.

The thirty-six male and female mice were divided into six groups of six mice each:

- Group 1 (Control): representing the nondiabetic group
- Group 2 (negative control): representing the diabetic group (HFD-STZ) untreated
- Group 3 (positive control): representing the diabetic group (HFD-STZ) treated orally with metformin at a dose of 300 mg/kg
- Group 4: representing the diabetic group (HFD-STZ) treated orally with the aqueous extract at a dose of 200 mg/kg
- Group 5: representing the diabetic group (HFD-STZ) treated orally with methanolic extract at a dose of 200 mg/kg
- Group 6: representing the diabetic group (HFD-STZ) treated orally with ethanolic extract at a dose of 200 mg/kg

Body weight and blood sugar were measured weekly for 1 month of treatment.

#### 2.5.2. Determination of Hematological and Biochemical Parameters

After 30 days of treatment, blood samples were taken from the jugular vein using capillary tubes containing ethylenediamine tetraacetic acid (EDTA) (anticoagulant). The following hematological parameters were examined in the blood samples collected: total hemoglobin (HGB), red (RBC), and white (WBC), and platelets were counted using a fully automated analyzer (Architect c8000, Clinical Chemistry System, Chicago, IL, UNITED STATES). Serum levels of aspartate aminotransferase (AST), alanine aminotransferase (ALT), urea, creatinine, cholesterol, triacylglycerols (TG), high-density lipoprotein (HDL), and low-density lipoprotein (LDL) were determined by the same analyzer.

#### 2.5.3. Statistical Analysis

Data were expressed as mean ± SEM. Statistical analysis and comparison of means were evaluated by one-way analysis of variance (ANOVA). The differences were considered statistically significant at *P* < 0.05. The analysis was performed with GraphPad Prism 6.

## 3. Results

### 3.1. Antihyperglycemic Activity

#### 3.1.1. Inhibitory Activities of *α*-Amylase and *α*-Glucosidase

Extracts of *E. guttatum* were tested for their inhibitory effects on *α*-amylase and *α*-glucosidase *in vitro*. The three extracts were examined at different concentrations of *α*-amylase and *α*-glucosidase and they were compared to the reference molecule acarbose (Figure 1). The three extracts had a significant inhibitory effect (*P* < 0.05) on *α*-amylase with a better effect presented by the methanolic extract of *E. guttatum* (EGM) with IC_50_ of 479.20 ± 0.81 *μ*g/mL (Table 1). On the other hand, the ethanolic extract of *E. guttatum* (EGE) of IC_50_ = 98.5 ± 0.81 *μ*g/mL showed a significantly (*P* < 0.05) greater effect than that of the aqueous extract of *E. guttatum* (EGA) (IC_50_ = 781.30 ± 0.54 *μ*g/mL). Thus, the extracts and the acarbose showed significant inhibitory activity (*P* < 0.05) on the *α*-glucosidase enzyme. All three extracts showed an inhibitory effect greater than that of acarbose. For IC_50_ values, EGA (4.88 ± 1.42 *μ*g/mL), EGM (3.67 ± 0.87 *μ*g/mL) and EGE (8.62 ± 0.90 *μ*g/mL) makes the IC_50_ of acarbose 18.01 ± 2.00 *μ*g/mL.

#### 3.1.2. Inhibitory Activities of Pancreatic Lipase

The study of the activity of *E. guttatum* extracts on pancreatic lipase is summarized in Table 2. The inhibitory activity of the extracts was evaluated at different concentrations (Figure 2). The reference compound Orlistat showed a superior inhibitory effect than extracts from *E. guttatum*. On the other hand, EGA, EGM, and EGE have shown an inhibitory effect against the enzyme pancreatic lipase. EGM with an IC_50_ = 31.6 ± 3.18 *μ*g/mL) had a significantly (*P* < 0.05) higher activity than that of EGA (IC_50_ = 84.7 ± 1.45 *μ*g/mL). In addition, EGE (48.05 ± 2.82) demonstrated a significantly (*P* < 0.05) lower effect compared to EGM.

#### 3.1.3. Oral Starch Tolerance in Normal Rats

As illustrated in Figure 3, the glycemia in all the groups was raised at 30 minutes after the starch load and then gradually decreased over the following hours. Acarbose at a dose of 50 mg/kg reduced postprandial hyperglycemia to 0.88 g/L after 120 min. The administration of extracts at a dose of 2.5 g/kg of starch (negative control) significantly induces hyperglycemia (1.26 g/L) in normal rats after 30 minutes. Thereafter, it is reduced to 0.97 g/L after 120 min. However, EGA, EGE, and EGM at 150 mg/kg after the starch load significantly reduced (*P* < 0.0001) the glycemia, respectively, to 0.79, 0.77, and 0.70 g/L after 120 min. Thus, the extracts decreased postprandial hyperglycemia compared to the negative control. The values of the area under the curve (AUC) of the acarbose as well as the extracts are lower than those of the negative control.

#### 3.1.4. Intestinal Absorption In Situ

The intestinal absorption of glucose evaluated in situ by the perfusion of the jejunal part of the rats is illustrated in Figure 4. Moreover, the amount of glucose absorbed from the jejunal part is 19.4 mg/10 cm/h. The perfusion of the EGA, EGE, and EGM at 200 mg/kg reduced glucose uptake compared to the control. The EGA significantly reduced (*P* < 0.001) the glucose absorption at 12.08 mg/10 cm/h compared to the control. The EGE significantly reduced (*P* < 0.001) the amount of glucose to 10.12 mg/10 cm/h, while the EGM caused a strong inhibition (*P* < 0.0001) of glucose to 7.4 mg/10 cm/h compared to the control phlorizin (0.1 mM), which inhibited significantly (*P* < 0.0001) the absorption of glucose at 8.6 mg/10 cm/h.

### 3.2. Antidiabetic Activity

#### 3.2.1. Fasting Blood Sugar

The effect of *E. guttatum* extracts and metformin on the blood sugar level for 30 days is summarized in Table 3. However, on the first day, a significant difference in blood sugar levels was observed between the groups of diabetic mice treated with the three extracts and metformin and the group of untreated diabetic mice with the normal group (*P* < 0.05). While there was no significant difference between the groups treated with the extracts and metformin compared with the untreated diabetic group (*P* > 0.05). Thus, after 30 days of treatment with *E. guttatum* extracts and metformin, blood sugar levels were significantly reduced compared to the untreated diabetic mouse group (*P* < 0.05).

The blood sugar levels of mice treated with metformin, EGE, and EGA are similar to those of normal mice. Likewise, the blood glucose value of mice treated with EGM is lower than that of normal mice.

#### 3.2.2. Body Weight

The change in body weight during 1 month of all groups of mice is shown in Table 4. At the start, there was a significant difference between diabetic mice treated with the extracts and metformin and the diabetic mice not treated with the normal mice (*P* < 0.05). Indeed, untreated diabetic mice gained weight (2.35%), while diabetic mice treated with metformin experienced body weight loss (3.38%). However, diabetic mice treated with EGM maintained a stable weight during the study period. And diabetic mice treated with EGA and EGE also experienced body weight loss. In addition, there was a significant difference between diabetic mice treated with EGA, EGM, and diabetic mice treated with metformin (*P* < 0.05). Likewise, there was not a significant difference between diabetic mice treated with EGA and EGM compared to untreated diabetic mice (*P* > 0.05).

#### 3.2.3. Hematological and Biochemical Parameters

The results of the effect of *E. guttatum* extracts on physiological function were examined on hematological and biochemical parameters (Table 5). Indeed, hemoglobin and platelets did not show a significant difference between the groups studied (*P* > 0.05). Also, there was a significant difference between the diabetic mice treated with extracts and metformin and the untreated diabetic mice (*P* < 0.05). In addition, the number of white blood cells in the diabetic mice treated with the extracts was higher than in normal mice. (*P* < 0.05) The number of white blood cells and hemoglobin increased in the group of untreated diabetic mice.

For cholesterol, TG and LDL were decreased in diabetic mice treated with EGA, EGM, EGE, and metformin compared to untreated diabetic mice, while the level of good HDL cholesterol increased in diabetic mice treated with EGA, EGM, EGE, and metformin. Moreover, for HDL, there was no significant difference between the diabetic mice treated with the extracts and metformin and with untreated mice (*P* > 0.05) whereas, for LDL, there was a significant difference between diabetic mice treated with extracts and metformin and untreated diabetic mice and normal mice (*P* < 0.05).

Regarding the hepatic profile, the ALT level in diabetic mice treated with the extracts is lower compared to diabetic mice treated with metformin. In addition, there was not a significant difference between groups for ALT (*P* > 0.05). Thus, untreated diabetic mice represent the highest rate of AST. Likewise, the AST level in diabetic mice treated with metformin is statistically similar to that of normal mice (*P* > 0.05).

For the renal profile, the creatinine level in normal mice and diabetic mice treated with the extracts and metformin is almost equal (*P* > 0.05). In addition, the urea level in diabetic mice treated with the extracts and metformin is lower compared to normal mice as well as untreated diabetic mice. Thus, there was a significant difference between the diabetic mice treated with the extracts and metformin and the untreated diabetic mice (*P* < 0.05).

## 4. Discussion

*α*-Amylase and *α*-glucosidase are the primary digestive enzymes involved in the catabolism of polysaccharides into easily absorbed simple carbohydrates [20]. However, this work contributed to studying the effect of *E. guttatum* on antidiabetic activity *in vitro* and *in vivo*. According to the results obtained, EGA, EGE, and EGM showed interesting *in vitro* inhibitory effects of *α*-amylase and *α*-glucosidase. Indeed, EGM exhibited the best inhibitory power on *α*-amylase and *α*-glucosidase with IC_50_ = 479.20 ± 0.81 *μ*g/mL and IC_50_ = 3.67 ± 0.87 *μ*g/mL, respectively. Therefore, these results are consistent with those of Sodik and Salamet [21], who worked on another Geraniaceae species (*E. collinum*). Their study revealed that the 50% aqueous-ethanolic extract of the root part exhibited potent *α*-glucosidase inhibitory activity, with an IC_50_ value of 0.09 *μ*g/mL. Polyphenols and flavonoids in plant extracts have been reported to be the main inhibitors of enzymes and glycosylated flavonoids, and these derivatives promote glucose blocking due to the hydroxyl group (OH) at C_3_ and the double bond between C_2_ and C_3_ of the C cycle of flavonoids [22]. Blocking the enzyme *α*-glucosidase helps with gastric evacuation, causes satiety, and results in weight loss in obese people [23].

Likewise, among the main enzymes in the digestion of lipids, pancreatic lipase breaks down triglycerides into free fatty acids and glycerol. Lipase inhibition remains among the most useful therapeutic approaches for diseases associated with lipid disorders, namely, obesity [24]. Orlistat is among the drugs most commonly used to inhibit lipase. It blocks about 30% of the absorption of fat of exogenous origin, but it has harmful effects such as diarrhea, greasy spots, abdominal cramps, gas, and fecal urgency [25]. Since antiquity, natural resources have occupied an important place. Currently, scientific research is interested in approving these therapeutic effects and enhancing them. In our study, the root extracts of *E. guttatum* significantly inhibited pancreatic lipase *in vitro*. EGA showed enzyme inhibition with IC_50_ = 84.7 ± 1.45 *μ*g/mL, EGM with IC_50_ = 31.6 ± 3.18 *μ*g/mL, and EGE with 48.05 ± 2.82 *μ*g/mL. According to the literature, bioactive compounds, mainly polyphenols, flavonoids, terpenoids, and other plant bioactive compounds, may be responsible for this effect [26]. On the other hand, the inhibitory activity of extracts on digestive enzymes can be explained by the type of extractant solvent. In this study, the methanolic extract is the most active, followed by ethanolic and aqueous extracts [25].

Also, we studied the effect of *E. guttatum* on postprandial hyperglycemia. All three extracts on oral starch tolerance reduced blood sugar levels in normal rats. The results also revealed that oral administration of EGM gave a better reduction in hyperglycemia. However, the activity of plant extracts could be associated with extra-pancreatic and pancreatic secretions [18]. In addition, the results demonstrated that the extracts accelerated the inhibition of intestinal absorption of glucose *in situ* like the reference molecule phlorizin. In addition, phlorizin, isolated from the plant *Pyrus communis*, belongs to one of the classes of polyphenols. It is characterized by its action of blocking the intestinal receptor SGLT1, evacuating glucose in the urine to decrease the reabsorption of glucose in renal epithelial cells and to improve blood sugar in diabetics [26]. These results can be explained by the fact that the extracts reduce glucose transport *via* inhibition of SGLT glucose transporters. Thus, these results corroborate the *in vitro* studies.

On the other hand, chronic administration of extracts of *E. guttatum* in diabetic mice resulted in body weight loss, which could be explained by the lipid-lowering activity of *E. guttatum*. In addition, we observed that the blood glucose level in mice rendered diabetic by HFD-STZ was increased. This elevation can be explained by the deterioration of the beta cells of the islets of Langerhans by STZ, causing insulinemia and insulin resistance to glucose and therefore an increase in blood sugar [27].

A high consumption of fats of exogenous origin will increase the oxidative capacity of fatty acids, reducing the use of glucose by insulin in the liver and skeletal muscle, resulting in insulin resistance in diabetics [28]. Insulin resistance results in decreased receptor substrate tyrosine phosphorylation (IRS), promoting insulin-activating signals [29]. The lipid profiles such as LDL, TG, and TC in the mice subjected to HFD-STZ were increased with a decrease in the HDL lipid level. The increased liver profiles, namely AST and ALT, are caused by leakage into the cytosol, inducing inflammation and necrosis of liver cells [28]. The increase in renal markers is an indicator of the development of diabetic nephropathy, causing osmotic diuresis and a reduction in the volume of extracellular fluid [30]. Our results showed that the treatment of diabetic mice with extracts of *E. guttatum* (200 mg/kg) reduced serum levels and protected against liver and kidney damage caused by HFD and STZ. Thus, it is suggested that the antidiabetic and antihyperlipidemic mechanisms could be due to the antioxidant activity of this plant. Indeed, studies have confirmed the richness of the extracts of *E. guttatum* in phenolic compounds. It has also been shown to have antioxidant activity by DPPH, H2O2, and xanthine oxidase assays [30, 31].

Overall, *Erodium* species contain many natural therapeutic agents, so *Erodium* species have been reported to be a rich source of natural antioxidants and phenolic compounds such as tannins (gerannin, dehydrogeraniin, and corrilagin) and flavonoids (isoquercetin, hyperin, and rutin) [12]. These observed results can be explained by the synergistic effect of various phenolic compounds contained in the plant, which may be responsible for these interesting therapeutic effects [32]. In addition, several scientific studies have demonstrated the antidiabetic power of natural resources [33]. For example, rutin has been confirmed to induce a reduction in the absorption of carbohydrates by the small intestine, the suppression of tissue gluconeogenesis, and the formation of sorbitol, reactive oxygen species, and product precursors that advance glycation endpoints [34]. Hyperine repairs pancreatic islet function and increases glycolysis [35]. Isoquercetin has shown an antihyperglycemic effect [36]. However, chemical compounds have become an alternative source of synthetics [37]. Therefore, the extracts of *E. guttatum* have strong antidiabetic and antihyperlipidemic activities and can be used as an alternative therapeutic approach to synthetic molecules for the prevention and treatment of diabetes mellitus.

## 5. Conclusion

*E. guttatum* extracts had an inhibitory effect on the digestive enzymes *α*-amylase, *α*-glucosidase, and lipase. Thus, they were found to have postprandial antihyperglycemic activity in normal rats. Also, they were able to lower blood sugar and restore the biochemical profile in mice made diabetic by HFD-STZ. However, other *in vivo* antidiabetic pathways need to be elucidated to understand their mode of action. As well as phytochemical studies must be addressed in order to identify the bioguided principles responsible for these effects.

## Figures and Tables

**Figure 1:** Percentage inhibition of *α*-amylase and *α*-glucosidase at different concentrations of *E. guttatum*. EGA: aqueous extract of *Erodium guttatum;* EGM: methanolic extract of *Erodium guttatum*; EGE: ethanolic extract of *Erodium guttatum.*

**Figure 2:** Percentage inhibition of pancreatic lipase at different concentrations of *E. guttatum*. EGA: aqueous extract of *E. guttatum;* EGM: methanolic extract of *E. guttatum*; EGE: ethanolic extract of *E. guttatum.*

**Figure 3:** Effect of *E. guttatum* extracts on glucose plasma levels after starch loading in normal rats (a) and with presentation in the area under the curve (b). The values are mean ± SEM (*n* = 6). ^*∗∗∗*^*P* < 0.001; ^*∗∗∗∗*^*P* < 0.0001 compared with normal controls. Ns = not significant to the normal controls. EGA: aqueous extract of *E. guttatum*; EGM: methanolic extract of *E. guttatum*; EGE: ethanolic extract of *E. guttatum*; AUC: area under the curve.

**Figure 4:** Effect of extracts of *E. guttatum* on intestinal glucose absorption by perfusion of the jejunal segment of rats with the perfusion solution containing glucose (1 g/L) and the extract at a dose (200 mg/kg). Data are mean ± SEM (*n* = 6). ^*∗∗*^*P* < 0.01; ^*∗∗∗*^*P* < 0.001; ^*∗∗∗∗*^*P* < 0.0001 compared with normal controls. EGM: methanolic extract of *E. guttatum*; EGE: ethanolic extract of *E. guttatum*; EGA: aqueous extract of *E. guttatum.*

**Table 1:** IC_50_ values of EGA, EGM, and EGE extracts on *α*-amylase and *α*-glucosidase inhibition.

	*α*-Amylase	*α*-Glucosidase
EGA	781.30 ± 0.54^*∗∗∗∗*^	4.88 ± 1.42^*∗∗*^
EGM	479.20 ± 0.81^*∗∗∗∗*^	3.67 ± 0.87^*∗∗*^
EGE	498.5 ± 0.81^*∗∗∗∗*^	8.62 ± 0.90^*∗∗*^
Acarbose	44.75 ± 0.54	18.01 ± 2.00

Values are mean ± SEM (*n* = 3). ^*∗∗*^*P* < 0.01, ^*∗∗∗*^*P* < 0.001, and ^*∗∗∗∗*^*P* < 0.0001. EGA: aqueous extract of *Erodium guttatum;* EGM: methanolic extract of *E. guttatum*; EGE: ethanolic extract of *E. guttatum.*

**Table 2:** IC_50_ values of EGA, EGM, and EGE extracts on lipase inhibition.

	Lipase
EGA	84.7 ± 1.45^*∗∗∗∗*^
EGM	31.6 ± 3.18^*∗∗∗*^
EGE	48.05 ± 2.82^*∗∗∗∗*^
Orlistat	12.55 ± 4.17

Values are mean ± SEM (*n* = 3). ^*∗∗∗*^*P* < 0.001 and ^*∗∗∗∗*^*P* < 0.0001. EGA: aqueous extract of *E. guttatum;* EGM: methanolic extract of *E. guttatum*; EGE: ethanolic extract of *E. guttatum.*

**Table 3:** Effects of *E. guttatum* extracts on fasting blood sugar in mice made diabetic by HFD-STZ.

Fasting blood sugar (mg/dL)		
	1 st day	30 days
Control normal	94.54 ± 15.32	110.42 ± 21.09
Diabetic control (STZ-HFD)	239.75 ± 26.42^*∗∗∗∗*^ns	295.1 ± 12.38††††ns
Diabetic + metformin (300 mg/kg)	253.17 ± 29.47^*∗∗∗∗*^ns	104.67 ± 4.08####ns
Diabetic + EGA (200 mg/kg)	250.33 ± 11.23^*∗∗∗∗*^ns	102.41 ± 4.22####ns
Diabetic + EGM (200 mg/kg)	236.02 ± 20.12^*∗∗∗∗*^ns	98.3 ± 12.6####ns
Diabetic + EGE (200 mg/kg)	253 ± 29.3^*∗∗∗∗*^ns	100.15 ± 29.14####ns

Values are mean ± SEM (*n* = 8). ^*∗∗∗∗*^*P* < 0.0001 compared to the normal control group. ^####^*P* < 0.0001 compared to the diabetic control group (HFD-STZ). ^††††^*P* < 0.0001 compared to the diabetic + metformin. Ns = not significant to the diabetic + metformin or diabetic control group (HFD-STZ) or normal control. EGA: aqueous extract of *E. guttatum;* EGM: methanolic extract of *E. guttatum*; EGE: ethanolic extract of *E. guttatum.* HFD: high-fat diet. STZ: streptozotocin. ^*∗∗∗*^present only statistical difference between results. They are explained by ^*∗∗∗∗*^*P* < 0.0001.

**Table 4:** Effects of *E. guttatum* extracts on body weight in mice made diabetic by HFD-STZ.

Body weight (g)		
	Initial weight	Final weight
Control normal	25.11 ± 4.18	29.53 ± 1.02
Diabetic control (STZ-HFD)	35.23 ± 1.87^*∗∗*^	36.08 ± 3.18^*∗∗∗∗*^†††
Diabetic + metformin (300 mg/kg)	33.3 ± 2.07^*∗*^ns	32.21 ± 0.7###ns
Diabetic + EGA (200 mg/kg)	35.12 ± 1.49^*∗∗*^ns	34.3 ± 1.11^*∗∗∗*^†ns
Diabetic + EGM (200 mg/kg)	34.61 ± 2.07^*∗∗*^ns	34.21 ± 1.04^*∗∗∗*^†ns
Diabetic + EGE (200 mg/kg)	34.75 ± 1.83^*∗∗*^ns	33.32 ± 1.2^*∗∗*^#

The values are the mean ± SEM (*n* = 6). ^*∗*^*P* < 0.05, ^*∗∗*^*P* < 0.01, ^*∗∗∗*^*P* < 0.001, and ^*∗∗∗∗*^*P* < 0.0001 compared to the normal control group. #*P* < 0.05 and ###*P* < 0.001 compared to the diabetic control group (HFD-STZ). †*P* < 0.05 and †††*P* < 0.001 compared to the diabetic + metformin. Ns = not significant to the diabetic + metformin or diabetic control group (HFD-STZ). EGA: aqueous extract of *E. guttatum;* EGM: methanolic extract of *E. guttatum*; EGE: ethanolic extract of *E. guttatum.*

**Table 5:** Effects of *E. guttatum* extracts on hematological and biochemical parameters in mice made diabetic by HFD-STZ.

	Normal control	Diabetic control (STZ-HFD)	Diabetic + metformin (300 mg/kg)	Diabetic + EGA (200 mg/kg)	Diabetic + EGM (200 mg/kg)	Diabetic + EGE (200 mg/kg)
*Hematology*						
WBC (10^−3^/*μ*L)	4.23 ± 0.89	21.31 ± 3.69^*∗*^^†^^*∗*^	10.43 ± 5.43#ns	9.22 ± 1.89^#^ns	7.86 ± 5.37^##^ns	7.33 ± 2.1^##^ns
RBC (10^−6^/*μ*L)	6.87 ± 0.02	8.36 ± 0.59 ns	7.84 ± 0.21 ns	9.90 ± 0.97^*∗∗∗*^†ns	8.88 ± 0.62^*∗*^ns	9.18 ± 0.65^*∗∗*^ns
HGB (g/dL)	11.25 ± 0.49	14.32 ± 1.27 ns	12.93 ± 0.98 ns	14.22 ± 1.35 ns	13.03 ± 0.55 ns	13.07 ± 0.66 ns
PLT (10^−3^/*μ*L)	508.00 ± 89.7	516.75 ± 93.11 ns	534.3 ± 51.18 ns	766.3 ± 339.9 ns	284.3 ± 103.2 ns	750 ± 232.1 ns

*Lipid profile*						
Cholesterol (g/L)	0.7 ± 0.01	3.48 ± 0.25^*∗∗∗∗*^	0.46 ± 0.17^*∗∗∗∗*^ns	1 ± 0.56^*∗∗∗∗*^ns	1.33 ± 0.19^*∗∗∗∗*^^#^ns	1.15 ± 0.16^*∗∗∗∗*^ns
TG (g/L)	0.83 ± 0.31	2.3 ± 0.26^*∗*^^††^	0.41 ± 0.16 ns^##^	1.77 ± 0.83^†^ns	2.2 ± 0.34^*∗*^^††^ns	1.59 ± 0.66 ns
HDL (mMol/L)	0.36 ± 0.06	0.14 ± 0.04 ns	0.21 ± 0.05 ns	0.49 ± 0.15^#^ns	0.4 ± 0.21 ns	0.46 ± 0.08^#^ns
LDL (g/L)	0.01 ± 0.001	0.26 ± 0.05^*∗∗∗*^	0.21 ± 0.09 ns^*∗∗*^	0.06 ± 0.01^##†^ns	0.14 ± 0.02 ns^*∗*^^#^	0.14 ± 0.01 ns^*∗*^^#^

*Liver function*						
AST (UI/L)	121.65 ± 5.28	266.17 ± 13.44 ns	118.33 ± 33.26 ns	176.5 ± 51.61 ns	483 ± 162.6^*∗∗∗*^^#†††^	218.5 ± 13.43 ns
ALT (UI/L)	39.27 ± 3.6	127.67 ± 12.5^*∗*^ns	84.66 ± 17.62 ns	55.33 ± 25.0 ns	70.33 ± 52.5 ns	61.5 ± 29.8 ns

*Renal function*						
Urea (g/L)	0.59 ± 0.07	0.62 ± 0.12 ns	0.43 ± 0.09 ns	0.34 ± 0.11 ns	0.51 ± 0.24 ns	0.35 ± 0.08 ns
Creatinine (mg/L)	3.78 ± 0.27	7.70 ± 1.49^*∗∗∗*^^†††^	4.18 ± 0.22^###^ns	3.30 ± 0.28^####^ns	4.1 ± 0.69^###^ns	3.43 ± 0.41^####^ns

The values are the mean ± SEM (*n* = 6). ^*∗*^*P* < 0.05, ^*∗∗*^*P* < 0.01, ^*∗∗∗*^*P* < 0.001, and ^*∗∗∗∗*^*P* < 0.0001 compared to the normal control group. ^#^*P* < 0.05, ^##^*P* < 0.01, ^###^*P* < 0.001, and ^####^*P* < 0.0001 compared to the diabetic control group (HFD-STZ). ^†^*P* < 0.05, ^††^*P* < 0.01, and ^†††^*P* < 0.001 compared to the diabetic + metformin. Ns = not significant to the diabetic + metformin or diabetic control group (HFD-STZ). EGA: aqueous extract of *E. guttatum;* EGM: methanolic extract of *E. guttatum*; EGE: ethanolic extract of *E. guttatum.*

## Data Availability

The data used to support the findings of this study are included within the article.
